The article "Automatic Parking System Based on Improved Neural Network Algorithm and Intelligent Image Analysis" was retracted in 2023. Reasons: unreliable results or conclusions; concerns about the data; concerns about the peer review; concerns about the citations.

# Automatic Parking System Based on Improved Neural Network Algorithm and Intelligent Image Analysis

**DOI:** 10.1155/2021/4391864

**Published:** 2021-09-17

**Authors:** Yucheng Guo, Hongtao Shi

**Affiliations:** ^1^Qingdao Jimo District Administration Examination and Approval Service Bureau of Shandong Province, Qingdao, Shandong 266200, China; ^2^School of Science and Information Science, Qingdao Agricultural University, Qingdao, Shandong 266109, China

## Abstract

This research designs an intelligent parking system including service application layer, perception layer, data analysis layer, and management layer. The network system adopts opm15 system, and the parking space recognition adopts improved convolution neural networks (CNNs) algorithm and image recognition technology. Firstly, the parking space is occupied and located, and the shortest path (Dynamic Programming, DP) is selected. In order to describe the path algorithm, the parking system model is established. Aiming at the problems of DP low power and adjacent path interference in the path detection system, a method of combining interference elimination technology with enhanced detector technology is proposed to effectively eliminate the interference path signal and improve the performance of the intelligent parking system. In order to verify whether the CNNs system designed in this study has advantages, the simulation experiments of CNNs, ZigBee, and manual parking are carried out. The results show that the parking system designed in this study can control the parking error, has smaller parking error than ZigBee, and has more than 25.64% less parking time than ZigBee, and more than 34.83% less time than manual parking. In terms of parking energy consumption, when there are less free parking spaces, CNNs have lower energy consumption.

## 1. Introduction

With the rapid development of national economy, the living standard of Chinese residents has been greatly improved, the travel conditions are more diverse and fast, and the number of private cars is increasing year by year. At the same time, due to the relative lag of urban planning and construction, there is a huge gap in the demand for parking space, and the problems of parking and finding a car are becoming increasingly prominent, which increases the efficiency of private car travel. In addition, the problems such as imperfect parking system and irregular parking have a significant impact on the overall travel, parking, and pick-up of residents. The design and promotion of intelligent parking system which can solve these problems has become an urgent demand.

Parking management services need to achieve a variety of functions, mainly including parking information query, map route navigation, display and guidance of spare parking spaces, intelligent payment, and car locating system, involving multidisciplinary technology, including edge computing, image processing technology, smartphone application development technology, and deep learning algorithm [1–3]. At present, there are some parking management service products in the market, but their functions are not perfect. The existing technical problems are mainly divided into three categories: inaccurate positioning, limited scope of use, inaccurate vehicle information identification and feedback, and some problems in promotion and cost. This research mainly aims at the technical level and carries out a series of design and improvement. In terms of positioning technology, due to the weak and inaccurate positioning signals of traditional positioning systems such as Global Positioning System (GPS) and Beidou, the widely used positioning technologies include ultrasonic positioning, infrared positioning, Radio Frequency Identification (RFID) positioning, Wireless Fidelity (WiFi) Positioning, ZigBee positioning, and Bluetooth positioning [4]. The positioning principle is to cover the field by building a wireless signal and then receive the signal and locate the object. The existing indoor positioning models include BP neural network positioning model, WLAN positioning model, support vector machine model, ZigBee fuzzy clustering positioning model, etc. [5]. In this study, WiFi coverage is used to identify and locate the free parking spaces.

Many achievements have been made in the research of vehicle navigation function. The navigation system is usually divided into three parts: parking lot end, cloud end, and user end. The parking lot information is transmitted to the cloud end and read at the user end after calculation and processing [6]. The system types include navigation system based on path planning, auxiliary navigation system using tags for mobile robots, and guidance system based on neural network algorithm for vehicle trajectory prediction [7]. This study uses the improved neural network algorithm for path navigation. The research of auxiliary parking system is relatively early, from the intelligent auxiliary parking system based on optical projection, to the 3D reconstruction automatic detection parking system, and the parking space monitoring system based on filter and local binary mode; now it can basically meet the needs of users [8]. Image recognition technology has also been greatly developed in recent years, such as parking space occupancy recognition technology based on C4.5 algorithm, Open Source Computer Vision Library (OpenCV) graphics processing technology, etc. [9]. This topic studies some image recognition technology and positioning technology, explores its existing application results, and optimizes its application mechanism. In view of the lack of accuracy and real time of current recognition technology, this study uses You Only Look Once (YOLO) improved model for image feature extraction and recognition, in order to improve its recognition efficiency and accuracy.

## 2. Establishment of Parking Space Recognition System Based on Improved Neural Network Algorithm

### 2.1. Overall Framework Design of Parking System

The parking system designed in this study is mainly divided into two parts: server part and data analysis part, including service application layer, perception layer, data analysis layer, and management layer [10]. The function of the service layer is that users can obtain some relevant information such as the number of cars in the parking lot, the entrance and exit of the parking lot, the estimated parking time, and so on, through the handheld terminal. At the same time, it also has the distance navigation function, which can plan the optimal path to the entrance of the parking lot and record the location information and parking time of the parking lot. The main function of the front-end perception layer is information transmission. The specific working principle is to obtain the recognition image of the parking space through the shooting function, recognize the coordinate information of the target parking space, and upload the information to the intelligent terminal. Combined with the positioning and navigation system of the intelligent terminal, the information is judged and analyzed, and the path is calculated. Cloud service layer, also known as data analysis layer, analyzes and calculates the obtained data by building a distributed cluster. In this study, the improved neural network algorithm and image recognition technology convolution neural network algorithm are used to analyze and process the data [11]. The main function of management is to manage, monitor, and maintain all levels. The system framework is shown in Figure 1.

The network system of parking system is opm15 system, which is composed of multiple network intelligent terminals with sensing ability, processing ability, and wireless communication performance, and can realize the interconnection communication between objects and between objects and networks [12]. Nodes in omp15 network can also be used as relay signals of other base stations to dynamically use network resources. The circuit connection diagram is shown in Figure 2.

It can be seen from Figure 2 that the power supply voltage of opm15 module is 3.3 V, the magnetic bead device with anti-high-frequency interference is set, and the reset I/O is set, which can send reset command and reset with one key. Receive External Data (RXD) and Transmit External Data (TXD) serial port can realize the communication of single chip microcomputer, as a terminal or router, and can also realize the communication of Personal Computer (PC), as a data communication acquisition and processing module.

### 2.2. Parking Space Recognition Technology Based on Convolution Neural Network Algorithm

The first step of automatic parking is to detect, identify, and locate the free parking space in the parking lot to get the real-time occupancy information. In this study, CNNs algorithm is used to extract the features of the collected parking image, identify the vehicle target, and then judge the parking occupancy [13]. The specific process is shown in Figure 3.

The feature extraction and recognition process is shown in Figure 3. The algorithm adopted by the feature extractor is the multilayer CNNs algorithm. The feature extraction process is to extract the overall image features first and then create candidate regions [14]. As shown in the figure, CNNs feature extractor selects conv5 convolution layer in Visual Geometry Group (VGG16) network to output feature map and generate candidate region of interest (ROI). Then, ROI is combined with corresponding feature map to be clipped to form target feature block. After ROI pooling, feature blocks are transformed into fixed size and enter the full connection layer. Then they are classified and located in the full connection layer, and the classification and recognition results are obtained. CNNs model can accurately identify parking spaces, but the real-time performance is poor. This study will improve the convolutional neural network recognition model and establish a one-time deep learning framework integrating YOLO algorithm to improve the real-time performance of convolutional neural network model recognition [15]. The model architecture is shown in Figure 4.

As shown in Figure 4, the framework of the YOLO model is completed in one step. The position box regression is directly performed on the input image information, and the target classification is carried out. The real-time performance is very high. As can be seen from the figure, the feature extraction network integrated with YOLO algorithm is composed of a large number of 3*∗*3 convolution cores and 1*∗*1 convolution cores. The output result is an *n*-dimensional feature map with 32 times *s∗s* size under the original image, and the feature map will enter the target box prediction operation and category prediction operation. Since the objects identified are vehicles in the parking lot and belong to a single class, and the sample size is small, the model integrated with YOLO algorithm can carry out large sample and multiclass complex recognition, which increases the complexity and time of operation [16, 17]. In order to reduce the complexity and time of operation, the sampling method is optimized. By reducing the redundant part of the model, the network training process of the network model is effectively simplified. Finally, the purpose of reducing the amount of operation of the neural network system is achieved and the detection efficiency is significantly improved. The improvement of sampling method is shown in Figure 5.

In Figure 5, *s∗s* in *s∗s∗n∗*(4+1+1) represents the number of grids, that is, the width of the feature graph, *n* represents the number of prior frames, that is, the number of anchor frames, and the data in (4 + 1 + 1) represents the number of border coordinates, border confidence, and object categories. The original YOLO algorithm uses 32 times of output multiple. In order to reduce the model, this study uses 16 times of multidimensional output combined with the setting of multiple anchor points. The obtained parking lot image is calibrated to get the YOLO shown in Figure 5, which is not a real label. In the label setting process, it is necessary to predict and judge the coincidence degree between the target box and the real box. In this study, the union intersection (IOU) algorithm is used to set the label and determine the number of labels [18]. The process of IOU algorithm determining label is shown in Figure 6.

As shown in Figure 6, *B*_1_ is set as the prediction box, *B*_2_ is set as the real box, and all prediction boxes and real calibration boxes are traversed. When the ratio IOU between the intersection (*B*_1_∩*B*_2_) and Union (*B*_1_ ∪ *B*_2_) of the position box is greater than 0.5, the prediction value is set as the real value and displayed in the label tensor for iterative training of convolution network.

### 2.3. Establishment of Parking Space Recognition System Based on Convolution Neural Network Algorithm

After the vehicles in the parking lot are accurately identified, it is necessary to establish a parking lot model. It is necessary to judge the coordinates of the detected vehicles and compare with the prior parking space box to judge the parking space occupation, which is reflected in the parking lot model. See Figure 7 for parking space identification.

Figure 7(a) is a parking lot model. The parking space in the figure corresponds to a parking space in the real parking lot (Figure 7(b)). The parking space recognition system is equipped on the parking lot model. Through real-time data processing, we can intuitively see whether each parking space has been occupied on the model. If *P* is included in the parking space model, it means that the parking space has been occupied. If *P* is not included, it means that the parking space is vacant. In the figure, we can also see the entrance and exit of the parking lot, the coordinates of the parking space, and the route and distance from the entrance and exit. The parking space recognition system based on the improved neural network algorithm is established.

## 3. Establishment of Vehicle Direct Path Detection System

### 3.1. Path Detection Interference Signal Elimination Technology

The communication network layer of this study is built by self-organizing network technology, which is divided into three parts: intelligent terminal, gateway, and handheld terminal. The user's handheld terminal needs to update the information in real time through the gateway and wireless communication system to keep the vehicle mobile data reflected in the handheld terminal in real time. The positioning performance of wireless communication system will be affected by external interference in the actual use process, which will affect the accuracy of the direct path signal, including the length, angle, and arrival time of DP, and even be difficult to distinguish and identify [19]. The interference is shown in Figure 8.

In Figure 8(a), adjacent road force signal interferes with DP signal, and DP signal received in Figure 8(b) is very weak. When the line of sight is obstructed, the path with the strongest signal selected may not be the optimal path. In the above two cases, direct path signal is difficult to be correctly identified. In this study, the multiprotocol label switching (MPLR) algorithm is used to eliminate the interference signal of the path outside DP. See the following formula for specific operation [20]:

(1) $$\begin{array}{c} x\left[n\right]=\sum_{k=0}^{N-1}X_{k}e^{j\left(2\pi kn/N\right)}, \end{array}$$

where *x*[*n*] represents the preamble transmitted in discrete time domain and *X*_*k*_ represents the preamble transmitted in *K* subcarrier segment. The expression of multipath channel *h*(*t*) is shown as follows:

(2) $$\begin{array}{c} h\left(t\right)=\sum_{\mu =0}^{N_{p}-1}a_{\mu }\delta \left(t-\tau_{\mu }\right), \end{array}$$

where *a*_*μ*_ is the complex channel gain of each path, *τ*_*μ*_ is the multidirectional transmission time (MTT) of the path, and *N* is the total number of paths. The expression of signal function from multipath channel to baseband is shown as follows:

(3) $$\begin{array}{c} y\left(t\right)=x\left(t\right)*h\left(t\right)+w\left(t\right), \end{array}$$

where *x*(*t*) is the baseband signal sent through the digital to analog converter (DAC), *w*(*t*) is the zero mean pseudo-Gaussian white noise;^*∗*^ represents convolution operation. The correlation function between the received signal *y*(*t*) and the leading signal is expressed by *C*. The expression of the function is shown as follows:

(4) $$\begin{array}{c} C\left[m\right]=\sum_{n=0}^{N-1}\bar{x\left(n\right)}y\left[m+n\right], \end{array}$$

where $\bar{\left(•\right)}$ represents complex conjugate and *m* represents the time index of *C*. In the case of multipath interference, the modified function of multipath channel is expressed as follows:

(5) $$\begin{array}{c} h^{\prime }\left(t\right)=\sum_{\mu \in O}\frac{a_{\mu }}{\zeta_{\mu }}\delta \left(t-\tau_{\mu }\right). \end{array}$$

where *O* is the path index set of traversing obstacles and *ζ*_*μ*_ is the transmission loss. There are two uncertain factors in formula (5), which affect the accuracy of the detection signal. One is the interference of adjacent paths, and the other is that the path delay time is not an integral multiple of the sampling time *T*_*s*_, which is missed in the sampling. The path detection method of interference cancellation can be realized by estimating the strong path MTT in the subsamples [21]. The MPLR algorithm is used to estimate MTT [22]. The specific expression is shown as follows:

(6) $$\begin{array}{c} \left\{\hat{\sigma },\hat{\varepsilon }\right\}=\arg\underset{\hat{\sigma },\hat{\varepsilon }}{\max}\frac{{\left|{\hat{h}}_{\hat{\theta }}\left(\hat{\varepsilon }\right)\right|}^{4}}{\left(1/\hat{\theta }\right)\sum_{m=0}^{\hat{\theta }-1}{\left|{\hat{h}}_{n}\left(\hat{s}\right)\right|}^{2}}, \end{array}$$

where $\hat{\theta }$ and $\hat{\varepsilon }$ represent the MTT of the sample cell, ${\hat{h}}_{\hat{\theta }}\left(\hat{\varepsilon }\right)$ represents the estimated time shifted channel, and the expression function is shown as follows:

(7) $$\begin{array}{c} \left|{\hat{h}}_{n}\left(\hat{\varepsilon }\right)\right|=\frac{1}{n}{\sum_{n}^{1}X_{k}}^{-{\tilde{y}}_{k}^{r}e^{j\left(2\pi k\hat{\varepsilon }/N\right)\left(2\pi kn/N\right)}}, \end{array}$$

where *r* is the time sample whose |*C*|^2^ exceeds the threshold *T* for the first time and ${\tilde{y}}_{k}^{r}$ represents the *k* − th frequency value in the discrete Fourier transform at the *N*-th point of the received time domain signal in the sample. *T* is the value of white Gaussian noise characteristics, which is expressed as follows:

(8) $$\begin{array}{c} T=\sqrt{-\ln\left(\frac{P_{FD}}{L}\right)2{\hat{\sigma }}_{F}^{2}}, \end{array}$$

where *P*_*FD*_ is the error detection probability, *L* is the length of the cyclic prefix, ${\hat{\sigma }}_{F}^{2}$ is the estimated noise variance, and ${\hat{\sigma }}_{F}$ is expressed as follows:

(9) $$\begin{array}{c} {\hat{\sigma }}_{F}=\sqrt{\frac{2}{\pi }}\left(\max\left\{{\left|C\right|}^{2}\right\}\right). \end{array}$$

The strong path MTT value measured by formulae (6)–(9) is the time shift function of *T* setting which will change according to the interference form of the filter. The form of interference is defined as *f*_tr_(*t*), and the sampling interval missing interference caused by delay time *t*_*p*_ can be expressed as formula (10).

(10) $$\begin{array}{c} {\hat{f}}_{l}\left[n\right]=\left\{\begin{array}{cc} \delta \left[n-\frac{t_{p}}{T_{s}}\right], & t_{p}=n\cdot T_{s},\\ f_{\text{tr}}\left(nT_{s}-t_{p}\right), & \text{others}. \end{array}\right. \end{array}$$

The amplitude adjustment of ${\hat{f}}_{l}\left[n\right]$ in formula (10) can be expressed as follows:

(11) $$\begin{array}{c} {\hat{f}}_{l2}\left[n\right]={\hat{f}}_{l}\left[n\right]\cdot \frac{{\hat{h}}_{\theta_{M}}\left(0\right)}{\max f_{l}\left[n\right]}, \end{array}$$

where ${\hat{h}}_{\theta_{M}}\left(0\right)$ is the maximum value. After modifying the estimated interference, ${\hat{h}}_{\theta_{M}}\left(0\right)$ convolutes with the transmitted signal, which can be expressed as follows:

(12) $$\begin{array}{c} y_{1}\left[n\right]=y\left[n\right]-{\hat{f}}_{l2}\left[n\right]*x\left[n\right]. \end{array}$$

*y*_1_[*n*] in formula (12) is the signal after interference cancellation. Strong path detection and interference cancellation are performed iteratively according to the above formula, and the result signal expression of the *i*-th iteration process is shown as follows:

(13) $$\begin{array}{c} y_{i}\left[n\right]=y_{i-1}\left[n\right]-{\hat{f}}_{l2}\left[n\right]*x\left[n\right]. \end{array}$$

During the iteration process, the MTT of the earliest path that exceeds the threshold is stored in a set until there is no strong path and the iteration process ends.

### 3.2. Enhanced Detector Algorithm and Its Fusion Improvement

The interference problem caused by low power of DP is solved by enhanced signal detector. The specific method is to use the product of *C* and ${\hat{h}}_{d}\left[n\right]={\hat{h}}_{n}\left(0\right)$ as a new function to observe DP more clearly and improve the performance of path detection. Constant false alarm rate (CFAR) algorithm is used to improve the performance of peak detection method, and *C* and ${\hat{h}}_{d}$ are used to improve the performance of DP detection [23]. The expression of algorithm function is shown as follows:

(14) $$\begin{array}{c} C\left[m\right]=Nh\left[m_{0}\right]+\sum_{\mu =1}^{N-1}D\left[m_{0}-m_{\mu }\right]h\left[m_{\mu }\right]+\sum_{n=1}^{N-1}w\left[m_{0}+n\right]\bar{x\left[n\right]}, \end{array}$$

*m*_*μ*_ is the MTT of the *μ* − th path, *h*[*m*_*μ*_] is the discrete time domain channel, and *h*[*m*_*μ*_] is the correlation between *x*[*n*] and *x*[*n*+*m*_0_ − *m*_*u*_]. The LS channel estimation method includes noise. See the following formula for details:

(15) $$\begin{array}{c} {\hat{h}}_{d}\left[m_{\mu }\right]=h\left[m_{\mu }\right]+g, \end{array}$$

where *g* is the error caused by *h*[*m*_*μ*_] and *P* can be defined as the product of *C* and ${\hat{h}}_{d}$. The logarithmic function of *P* can further improve the detection performance of DP and reduce the occurrence of missing detection events. However, the interference of the enhanced DP detector to the adjacent path is still difficult to eliminate, so this study will combine the interference elimination and enhanced path detection technology to further improve the detection performance of DP [24]. The intersection of the results obtained by the two techniques is the result of our algorithm, which is expressed as follows:

(16) $$\begin{array}{c} F_{C}=\min\left(F_{A}\cap F_{B}\right), \end{array}$$

where *F*_*C*_ is the final result of the algorithm, *F*_*A*_ is the result set of the interference elimination algorithm, and *F*_*B*_ is the result set of the enhanced path algorithm. Compared with the traditional technology, the path screened by the enhanced path detector can be distinguished from the noise, which may lead to performance difference [25]. The performance improvement of the algorithm is shown in Figure 9.

As shown in Figure 9, the cumulative distribution function (CDF) in four different environments is described. The absolute error median of the proposed algorithm is about 0.8 m, which has a significant improvement with the traditional algorithm of 2–5 m. It can be inferred that the algorithm combining interference elimination and enhanced path detection is feasible in indoor environment. The algorithm is embedded in the intelligent parking system and the simulation experiment platform is established. The operating environment of the platform is tomcat9.0, mysql6.4, and jdk8.0. The platform development tools are eclipse ad t26.7, MySQL client 15.0, and my eclipse17.0. The test management tool adopts MAT8.1.

## 4. Experiment and Results

### 4.1. Comparison of System Parking Error

In this study, a parking lot is selected, each parking space in the parking lot is covered with intelligent terminal cameras, and seven handheld terminals are set, of which four terminals are used for mobile, three terminals are used for parking management, and one gateway is set on both sides of the parking lot to ensure network communication. In addition, in order to compare the performance of the system designed in this paper more scientifically, in the same experimental environment, the ZigBee parking guidance system and the CNNs used in this paper are selected for comparative experiments, and the results are compared and analyzed. The parking error comparison of the two systems is shown in Figure 10.

Figure 10 shows the error comparison between the ZigBee system and the CNNs system in this paper. As can be seen from Figure 10(a), the *x*-axis errors of the two algorithms are very small and can be ignored. It can be seen from Figure 10(b) that both systems have certain *Y*-axis error. The error of CNNs system is relatively small, especially in the process of 0–25 seconds; ZigBee system has obvious negative error. In the process of 25–40 seconds, the negative error of ZigBee system decreases, while CNNs system produces positive error. In the whole process, the error of CNNs system is controlled between −5 cm and +5 cm, and the error of ZigBee system is controlled between −10 cm and +10 cm. As can be seen from Figure 10(c), both algorithms have body errors. In the early 5–10 s parking process, the CNNs error is small, and in the later 30–40 s parking process, the ZigBee algorithm error is small, and the overall body error is controlled at 3° Within.

### 4.2. Time-Consuming Comparison of Automatic Shutdown System

The time-consuming comparison experiment still uses ZigBee system to compare with the CNNs system in this paper. In addition, a complete artificial parking experiment without the assistance of intelligent system is added as a reference, by making it the control group [25]. The scenarios with 20, 40, 60, 80, 100, and 120 free parking spaces are selected as the experimental conditions of this experiment. Five simulation experiments are carried out under each experimental condition, and the average of the results is taken for comparative analysis. The parking process is divided into three stages. The first stage is the process of the entrance of the parking lot in the target parking space. The second stage is the process of finding the parking vehicle from the starting point. The third stage is the process of starting from the parking space to the exit of the parking lot. In the process of the simulation experiment, the state of the parking lot is consistent, and the target nodes are consistent, which fully ensures the consistency of the experimental conditions and the scientificity of the results. The results are shown in Figure 11.

As shown in Figure 11, when the number of free parking spaces in the parking lot is 20, the average time of five simulation experiments of CNNs is 9.1 seconds, the average time of ZigBee system is 14.7 seconds, and the average time of parking without intelligent system is 18 seconds. CNNs have a very significant time advantage. When there are 40 or 60 parking spaces, the parking time of CNNs is slightly shortened, the parking time of ZigBee system and manual parking is significantly shortened, and the parking time difference between CNNs and the other two situations is reduced. When there are 80, 100, and 120 free parking spaces, the parking time of CNNs is still significantly better than the other two cases, and the time gap is further narrowed. When there are 120 parking spaces left, CNNs parking time is 5.8 seconds, ZigBee parking time is 7.8 seconds, and manual parking time is 8.9 seconds. On the whole, the time consumption of CNNs intelligent parking navigation system is 25.64% less than that of ZigBee and 34.83% less than that of manual parking.

### 4.3. Energy Consumption Comparison of Automatic Parking System

ZigBee system and CNNs system are used for energy consumption experiment. Since no intelligent system is used for parking experiment; there is no phenomenon of system energy consumption, so the control group is deleted. The scenarios with 20, 40, 60, 80, 100, and 120 free parking spaces are selected as the experimental conditions of this experiment. Five simulation experiments are carried out under each experimental condition, and the average of the results is taken for comparative analysis. The simulation results are shown in Figure 12.

As shown in Figure 12, with the increase of the number of vacant parking spaces in the parking lot, the amount of information and calculation needed to be processed by the system increases, and the energy consumption will also increase. When there are 20 vacant parking spaces, the energy consumption of CNNs is 24 MW, ZigBee energy consumption is 46 MW, and that of CNNs is about 47.8% lower than ZigBee. With the increase of parking space, the energy consumption of both systems is increasing. When the number of vehicles reaches 120, the energy consumption of CNNs reaches 110 MW, ZigBee energy consumption is 101 MW, and CNNs is higher than ZigBee energy consumption by 8.1%. When the parking space is less, the energy consumption of CNNs is lower than that of ZigBee parking system. With the increase of parking space, the proportion of free parking spaces increases, and the energy consumption of CNNs exceeds ZigBee. The relationship between energy consumption and the ratio of spare space remains to be further studied.

## 5. Conclusion

This research designs the intelligent parking system for parking problem, including service application layer, perception layer, data analysis layer, and management layer. Among them, opm15 module is used as intelligent terminal in the network system to realize operation and network information transmission. The improved convolution neural network algorithm and image recognition technology are used to identify and locate parking space. Then, the vehicle license plate information is identified by using the improved model of YOLO model, then the parking system model is established, and the DP selection algorithm is described by the model. Because of the two problems in the path detection system, which are DP low power and strong signal interference of adjacent paths, a method combining interference elimination technology and enhanced detector technology is proposed to eliminate the interference path signal effectively. In order to verify the superiority of the designed CNNs system in this study, the simulation experiment is designed. The experimental comparison between CNNs and ZigBee and artificial parking is carried out. The results show that the control error of *x*-axis in parking error of the parking system designed in this study is close to 0, the *Y*-axis error is between −5 cm and +5 cm, and the body error is 3° within; compared with ZigBee, it has smaller parking error and has a significant advantage over ZigBee and manual parking time, with a time consumption of 25.64% less. In the parking energy consumption, when there is less free parking space, CNNs have lower energy consumption, and the system energy consumption increases when there are more free parking spaces, and ZigBee algorithm shows lower energy consumption. Overall, the intelligent parking system proposed in this study has the characteristics of small parking error, short time consumption, and low-energy consumption. In order to further reduce the system energy consumption and time required, the intelligent parking system proposed in this topic should be continuously optimized to build a more efficient and low-energy parking system for the situation of large parking space margin.

## Figures and Tables

**Figure 1:** Overall system framework design.

**Figure 2:** opm15 circuit diagram.

**Figure 3:** Feature extraction and recognition of convolution neural network.

**Figure 4:** YOLO model architecture.

**Figure 5:** Truth label diagram.

**Figure 6:** IOU calculation method.

**Figure 7:** Parking map. (a) Parking hypothesis map. (b) Parking space identification example map.

**Figure 8:** DP difficult to detect situation. (a) Interference from adjacent paths. (b) Low power DP.

**Figure 9:** Comprehensive performance comparison in various environments.

**Figure 10:** Comparison of system parking error. (a) Parking *X*-axis error. (b) Parking *Y*-axis error. (c) Parking body angle error.

**Figure 11:** Comparison of system consumption time.

**Figure 12:** Comparison of system energy consumption.

## Data Availability

The data used to support the findings of this study are available from the corresponding author upon request.

## References

[1] Anagnostopoulos T., Fedchenkov P., Tsotsolas N., Ntalianis K., Zaslavsky A., Salmon I. (2020). Distributed modeling of smart parking system using LSTM with stochastic periodic predictions. *Neural Computing & Applications*.

[2] Bai D., Lv X., Wang J., Wenjie Z. (2020). Application of directional transmission data technology for transmission lines. *Journal of Physics: Conference Series*.

[3] Gao J., Chen Y., Wei Y., Li J. (2021). Detection of specific building in remote sensing images using a novel YOLO-S-CIOU model. Case: gas station identification. *Sensors*.

[4] Hisung M., Reuss H.-C. (2021). Automated vehicle positioning system for inductive charging. *ATZ Worldwide*.

[5] Hurst-Tarrab N., Chang L., Gonzalez-Mendoza M., Hernandez-Gress N. (2020). Robust parking block segmentation from a surveillance camera perspective. *Applied Sciences*.

[6] Jingyu A., Jing W., Linan C. (2020). Control method of urban intelligent parking guidance system based on internet of things. *Computer Communications*.

[7] Kang I. B., Park J., Lee J., Lee Y., Lim C. (2020). Flower classification with modified multimodal convolutional neural networks. *Expert Systems with Applications*.

[8] Kessentini Y., Besbes M. D., Ammar S., Chabbouh A. (2019). A two-stage deep neural network for multi-norm license plate detection and recognition. *Expert Systems with Applications*.

[9] Kim G., Park J., Chung K. (2019). MQTT-based gateway system for auto-configuration of iot devices and services. *Journal of KIISE*.

[10] Kim J., Park M., Bae Y. (2020). A low-cost, high-precision vehicle navigation system for deep urban multipath environment using TDCP measurements. *Sensors*.

[11] Prasetyo B. A., Wahyu A. P., Suhendri S. (2021). Optimization of image processing techniques in developing of smart parking system. *Journal of Information Technology*.

[12] Iqbal R., Maniak T., Karyotis C. (2019). Intelligent remote monitoring of parking spaces using licensed and unlicensed wireless technologies. *IEEE Network*.

[13] Rahman A. (2021). Radio frequency identification based smart parking system using internet of things. *IAES International Journal of Robotics and Automation*.

[14] Shan S. L., Jiang M. S., Su C. H., Zhang L. (2020). Novel phase difference extraction method of FPP system based on DWT and OMP algorithm. *Optoelectronics Letters*.

[15] Sobeslav V., Horalek J. (2020). A smart parking system based on mini PC platform and mobile application for parking space detection. *Mobile Information Systems*.

[16] Song K., Wei L., Bao F. J. I., Wang Y., Huang Y., Yang L. (2016). Outage performance for heterogeneous cellular networks with interference cancellation. *Dianzi Yu Xinxi Xuebao/Journal of Electronics and Information Technology*.

[17] Tang J., Zhu Y., Huang Y., Peng Z.-R., Wang Z. (2019). Identification and interpretation of spatial-temporal mismatch between taxi demand and supply using global positioning system data. *Journal of Intelligent Transportation Systems*.

[18] Thu N. T., Layek M. A., Huh E. N. (2019). An effective vision-based self-navigation system for autonomous indoor vehicle. *KIISE Transactions on Computing Practices*.

[19] Varahram P., Mohammady S., Farrell R., John D. (2020). A crest factor reduction scheme with optimum spacing peak cancellation for intra-band non-contiguous carrier aggregated OFDM signals. *Wireless Personal Communications*.

[20] Xian J., Liu X. X., Tongwei Z., Qiming W. (2020). Robust data cleaning methodology using online support vector regression for ultra-short baseline positioning system. *The Review of Scientific Instruments*.

[21] Yang S., Ma W., Pi X., Qian S. (2019). A deep learning approach to real-time parking occupancy prediction in transportation networks incorporating multiple spatio-temporal data sources. *Transportation Research Part C: Emerging Technologies*.

[22] Yazdi H. A., Pourmina M. A., Haghbin A. (2021). A robust acquisition technique using CFAR adaptive thresholding in hybrid spread spectrum systems. *Wireless Personal Communications*.

[23] Zhang K., Polycarpou M. M., Parisini T. (2020). Enhanced anomaly detector for nonlinear cyber-physical systems against stealthy integrity attacks. *IFAC-PapersOnLine*.

[24] Zhou C., Wang H., Wang H., Bo Hu (2021). Three-dimensional asperity model of rough surfaces based on valley–peak ratio of the maximum peak. *Meccanica*.

[25] Лернер И. М. (2019). Capacity estimation of wireless communication systems based on the choice of the optimal complex frequency channel response. *Вестник Казанского Го*.

